# PSMA1, a Poor Prognostic Factor, Promotes Tumor Growth in Lung Squamous Cell Carcinoma

**DOI:** 10.1155/2023/5386635

**Published:** 2023-02-03

**Authors:** Zhao Liu, Wuping Wang, Yanwu Zhou, Linfeng Li, Wolong Zhou

**Affiliations:** ^1^Department of Thoracic Surgery, The Sixth Affiliated Hospital of Xinjiang Medical University, Urumqi, Xinjiang Uygur Autonomous Region 830002, China; ^2^Department of Thoracic Surgery, Xi'an International Medical Center Hospital, Xi'an, Shaanxi 710100, China; ^3^Department of Thoracic Surgery, Xiangya Hospital Central South University, Changsha, Hunan 410008, China

## Abstract

Lung squamous cell carcinoma (LUSC) has a poor clinical prognosis and lacks effective targeted therapy. This study is aimed at investigating the role of PSMA1 (proteasome subunit alpha type-1) in LUSC. The differential expression genes (DEGs) in LUSC were retrieved from The Cancer Genome Atlas (TCGA) by “edgR” algorithm and by “limma” R package. Then, the relationship between genes and overall survival (OS) was explored by the least absolute shrinkage and selection operator (LASSO) and multivariate Cox (multi-Cox) regression. Next, the PSMA1 expression in tissues of LUSC was detected by IHC, qRT-PCR, and western blot (WB). Moreover, the effects of PSMA1 on the proliferation and viability of LUSC cell were explored by cell counting kit 8 (CCK-8) assays, colony formation assays, and flow cytometry (FCM) analysis. All 4421 DEGs were screened by TCGA database, and 26 genes associated with OS were selected by multi-Cox. Based on TCGA database, PSMA1 was highly expressed in tissues of LUSC patients, and OS and FP of patients with PSMA1 overexpression were significantly lower than those of patients with low PSMA1 expression. Furthermore, PSMA1 knockdown significantly decreased the proliferation of LUSC cells and promoted the apoptosis of LUSC cells, and these effects were reversed by PSMA1 overexpression. The results of this project supported that PSMA1 might be a critical gene regulating the development of LUSC and has the potential to be explored as a prognostic biomarker of LUSC.

## 1. Introduction

Lung squamous cell carcinoma (LUSC), the second common histologic subtype of non-small-cell lung cancer (NSCLC), is associated with poor clinical prognosis and limited treatment progress [1]. Driver mutations are common in LUSC, a highly heterogeneous disease, and mutations have been identified in a large number of genes, such as TP53 and PIK3CA [2]. Even in the early stage of LUSC, LUSC has extremely high tumor mutation burden (TMB) with over 200 outward mutations in some cohorts [3]. TMB is associated with the development of LUSC, and TMB-associated genes can be used to predict the OS of LUSC [4]. The mutations in tumor protein p53 (TP53) and cyclin-dependent kinase inhibitor 2A (CDKN2A) accounted for over 81% genomic alteration in LUSC [5]. However, no regimens targeting these mutations have been approved for LUSC [6]. TCGA program has catalyzed systematic characterization of diverse genomic alterations underlying human cancers, which could be used to explore prognostic genes in LUSC.

PSMA1 is one of the 17 essential subunits of the 20S proteasome, a multicatalytic proteinase complex with a highly ordered ring-shaped core structure, which is relevant to the survival of MDS and AML cells and plays a critical role in multiple neoplasms [7]. PSMA1 has been reported to be a promising biomarker that could be used to screen and diagnose early-stage colon cancer [8]. PSMA1 has been reported to be highly expressed in breast cancer [3]. Another study revealed that circPSMA1 functions as a tumor promoter which can facilitate the tumorigenesis, metastasis, and immunosuppression of triple-negative breast cancer (TNBC) [9]. However, there are few studies on how PSMA1 acts as a prognostic factor in LUSC. In our study, bioinformatics analyses and LASSO model analyses were integrated to explore potential prognostic biomarker, and we also identified the mechanism of PSMA1 in LUSC.

## 2. Methods

### 2.1. Data Collection

The gene expression data from TCGA and GTEx were all Trans Per Million (TPM) normalized from the raw RNA-Seq data, which belongs to the UCSC Xena project based on a uniform pipeline (http://xena.ucsc.edu/). TIMER is a database that is capable of analyzing the clinical impact of different immune cells in diverse cancer types [10]. The relationship between the expression level of PSMA1 and progression of LUSC was also analyzed through the TIMER database (https://cistrome.shinyapps.io/timer). *P* < 0.05 was deemed statistically significant. UALCAN (http://ualcan.path.uab.edu/) is used to export results of gene expression and survival analysis based on TCGA [11]. In this work, UALCAN was performed to clarify the differential expression levels of PSMA1 in tumor and normal tissues. Survival analysis of the PSMA1 in LUSC tissue was conducted by the Kaplan-Meier plotter, an online database (http://kmplot.com/analysis), which is able to assess the correlation between the expression of genes (mRNA, miRNA, and protein) and survival [12].

### 2.2. The Construction of Multigene Signature Risk Score Model

Differential RNA expression between the LUSC group and normal group was identified by “edgR” algorithm and by “limma” R package [13]. The criteria for differential RNAs to be selected are adj.*P*.Val < 0.05 and |logFC(logFoldChange)| > 1. According to the detected prognostic genes, the significant signature associated with survival was further investigated by the LASSO regression model. Then, in order to filter out the independent prognostic factors from these robust genes, multi-Cox regression analysis was performed with the “survival” R-package.

### 2.3. Clinical Tissue Collection and Cell Culture

In this study, all specimens were collected by the Sixth Affiliated Hospital of Xinjiang Medical University, in compliance with institutional consent and Institutional Review Board (IRB) protocols (Approval No. LFYLLSC20190617-01). All 30 pairs of the samples were obtained with a diagnosis of LUSC. Our study was performed in accordance with appropriate data protection legislation and the provisions of the Declaration of Helsinki. Written informed consent was obtained from each patient for the use of tissue samples. Fresh tissues were dissected immediately after surgical removal from patients, flash frozen in liquid nitrogen, and stored at −80°C.

The human LUSC cell lines including LTEP-s, NCI-H596, NCI-H520 cells, and the normal lung cell line BEAS-2B were obtained from the National Infrastructure of Cell Line Resource (Beijing, China), and the cells were cultured in complete Dulbecco's modified Eagle's medium (DMEM) (Gibco, Grand Island, USA) supplemented with 10% fetal bovine serum (FBS) (Gibco, Grand Island, USA) and 1% penicillin/streptomycin (1 : 100) (Gibco, Grand Island, USA). The cells were preserved in a 5% CO_2_ humidified incubator at 37°C.

### 2.4. Plasmid Construction, shRNA, and Transfection

Following the manufacturer's instructions, the pHB-Basic vector (HANBIO, Shanghai, China) was used to subclone PSMA1. The PSMA1-overexpressed plasmid was selected with penicillin and verified by sequencing. Moreover, two lentivirus-mediated short hairpin RNAs (shRNAs) were used to silence PSMA1. The qRT-PCR was applied to examine the efficiency; shRNA-1 and shRNA-2 were recognized as the effective shRNAs. shRNA-1 and shRNA-2 were synthesized by RiboBio (Guangzhou, China). We use electrotransfection to transfect cells with PSMA1-overexpressed plasmid by a NEPA 21 electroporator (NEPA, Japan). LTEP-s and NCI-H596 were infected with lentivirus carrying PSMA1-overexpressed vector according to the manufacturer's instructions and then selected with 1 *μ*g/mL puromycin. The sequences of shRNAs are listed in Table 1.

### 2.5. Cell Counting Kit-8 (CCK-8) Assay

BEAS-2B, LTEP-s, NCI-H596, and NCI-H520 cells were plated into 96-well plates with a density of 3 × 10^4^ cells/well for 0 h, 24 h, 48 h, 72 h, and 96 h. Cell viability was detected by CCK-8 reagent (100 *μ*L/mL medium) with incubation for 2 h, and the absorbance was detected at 450 nm using a microplate reader (Molecular Devices, Silicon Valley, USA).

### 2.6. RNA Isolation and Reverse Transcription-Quantitative Polymerase Chain Reaction (RT-qPCR)

The RNAprotect Cell Reagent was applied to isolated total RNA. The qRT-PCR was performed by a QuantStudio™ 7 Flex Real-Time PCR System (Life Technologies, Loughborough, UK) and NovoStart®SYBR qPCR SuperMix Plus. The expression of PSMA1 was normalized against that of GAPDH using the 2^−*ΔΔ*Ct^ method and presented as mean ± SD of replicates. mRNA was reversed transcribed to synthesize cDNA according to the manufacturer's instructions through PrimeScript™ RT Reagent Kit (Takara, Japan) on an iCycler iQ system (Bio-Rad, USA). The primers for PSMA1 and GAPDH primers are shown in Table 2 [9].

### 2.7. Western Blot Analysis

The total protein was isolated by modified RIPA buffer (P0013B; Beyotime, Shanghai, China) and was quantitated by BCA Protein Assay Kit (P0010; Beyotime, Shanghai, China). Then, the total protein was separated by 10% sodium dodecyl sulfate-polyacrylamide gel electrophoresis (SDS-PAGE). Next, the proteins were transferred to polyvinylidene fluoride (PVDF) membranes and then blocked in 5% milk diluted with TBST for 1 h at room temperature and probed with primary antibodies, PSMA1 (Abcam, ab71720, 1 : 500) and *β*-actin (Abcam, ab119716, 1 : 1000), at 4°C overnight. Then, a secondary rabbit anti-rabbit antibody (1 : 1000) was used to incubate the membranes at the following day for 1 h at room temperature. The ImageJ software was used for quantitation of the immunoreactive bands.

### 2.8. Immunohistochemistry (IHC)

Before staining, paraffin sections (4 *μ*m thickness) were heated overnight at 60°C. The slides were washed with TBS (pH 7.4), and antigens were retrieved with Tris/borate/EDTA buffer (pH 8-8.5) by heating at 95°C for 8 min and boiling at 100°C for 1.5 h. Tissue sections were incubated with anti-PSMA1 antibody (1 : 400 dilution) in TBS containing 1% BSA at 37°C for 1 h. Antibody reaction was detected with the UltraView Universal DAB Detection Kit (Ventana). Hydrogen peroxide substrate and 3, 3′-diaminobenzidine tetrahydrochloride (DAB) chromogen were used to visualize the complex, because they could produce a dark brown precipitate which was able to be detected by light microscopy. In line with the average stain intensity, immunohistochemical was scored as follows: 3 for dark brown color, 2 for medium brown, 1 for weak brown, and 0 for no staining.

### 2.9. Colony Formation Assay

A total of 2 mL LTEP-s and NCI-H596 cells were plated by a density of 5 × 10^3^ each well into 6-well plates and cultured for two weeks. The cells were rinsed by PBS 3 times and fixed by methanol for 10 min. The aimed cells were stained with Giemsa dye and counted under a microscope.

### 2.10. Flow Cytometry

The percentage of apoptotic cells was both stained with fluorescein isothiocyanate- (FITC-) conjugated Annexin V and propidium iodide (PI) which is referred to the manufacturer's protocols. The cells were run on either a three-laser BD Canto-II or a four-laser BD LSRFortessa X-20, using FACS Diva software (BD Biosciences). Acquired data files were analyzed using FlowJo 10.01 (BD Biosciences).

### 2.11. Statistical Analyses

SPSS version 21.0 software was applied to analyze data. And the data comparison used unpaired Student's *t* test within the 2 groups for statistical significance. The Spearman correlation analysis and distance correlation analysis were conducted to calculate correlation coefficient. In order to assess whether the difference is statistically significant, the log-rank test was used in a calculated way. The difference is deemed to be significant, when the two-tailed *P* value must be <0.05.

## 3. Results

### 3.1. Identification of DEGs in LUSC Based on TCGA Database

DEGs for NSCLC were interpreted and identified by the “edgR” algorithm and the “limma” R package based on TCGA database. First, the “limma” R package was used to select differentially expressed genes according to the threshold of adjust *P* value < 0.05 and |log FC| > 1. A total of 4866 differential genes were obtained, including 2437 upregulated genes and 2429 downregulated genes (Figure 1(a)). Second, volcano plots listed in Figure 1(b) suggested that 4958 differentially expressed genes were screened by the edgR package based on the threshold of FDR < 0.05 and logFC > 1, which included 2930 upregulated genes and 2028 downregulated genes. The overlapping of genes between the results of the limma package and edgR package is shown in Figure 1(c). The results showed that 4421 genes were found in both the limma package and edgR package.

### 3.2. Identification of Prognostic Genes in LUSC Based on Machine Learning Model

The merge function in R was adopted to integrate the expression profiles of the 12,912 module genes with the corresponding 360 LUSC patients' survival time and status information. Notably, 40 genes associated with overall survival (OS) were then identified by uni-Cox analysis (Figure 2(a)). According to the characteristics of variable selection and regularization, LASSO regression (LASSO-Cox) was performed while fitting a generalized linear model (Figures 2(b) and 2(c)). Then, 26 genes associated with OS were selected by multi-Cox analysis (Figure 2(d)), including PSMA1 (HR (95%CI) = 1.93, P = 8.53 *e*^−06^).

### 3.3. Expression Level and Prognosis of PSMA1 in LUSC

In this study, the mRNA expression of PSMA1 in LUSC samples and normal samples was compared in the TIMER database (Figure 3(a)) and UALCAN database (Figure 3(b)), respectively. The results indicated that PSMA1 was highly expressed in tissues of LUSC patients. The KMplot platform was performed to explore the association between PSMA1 expression and the prognosis of LUSC. The results in Figures 3(c) and 3(d) showed that the OS rate and FP of patients with PSMA1 overexpression were significantly lower than those of patients with low PSMA1 expression. Thus, survival analysis revealed that PSMA1 overexpression was significantly connected with reduced OS and FP in LUSC patients. The above results revealed that high expression of PSMA1 was associated with poor prognosis in LUSC patients.

### 3.4. Exploration of the Expression of PSMA1 in Cells and Tissue

The expression of PSMA1 in 30 pairs of LUSC tissues and adjacent normal tissues was detected through qRT-PCR. As shown in Figure 4(a), PSMA1 expression was significantly increased in LUSC tissues compared with normal tissues. Moreover, western blot experiments suggested that PSMA1 protein was increased in LUSC tissues (Figure 4(b)). Expression of PSMA1 was detected by IHC, and the results showed that the number of PSMA1-positive cells in LUSC tissues was significantly higher than that in normal tissues (Figure 4(c)). No statistical differences were observed between PSMA1 expression, gender, and age. Evidently, the high expression of PSMA1 was distinguished with the low expression of PSMA1 in TNM stage, pathological grading, and smoking (Table 3).

The expression level of PSMA1 was further validated in LTEP-s, NCI-H596, and NCI-H520 cells. The qRT-PCR results suggested that the mRNA expression of PSMA1 in LUSC cells was abnormally increased compared with that in the control group (Figure 4(d)). The results in Figure 4(e) showed that the protein expression of PSMA1 was also higher than that of normal tissue. These results suggested that the expression of PSMA1 was increased in both cells and LUSC patients' tissue.

### 3.5. PSMA1 Regulates Proliferation and Cell Viability of LUSC

In order to investigate the potential biological functions of PSMA1 in LUSC, the expression of PSMA1 was silenced through transfecting LTEP-s and NCI-H596 cells with shPSMA1-1# and shPSMA1-2#. PSMA1 overexpression was achieved by transfecting LTEP-s and NCI-H596 cells with vector-PSMA1. The expression level of PSMA1 was increased in the vector-PSMA1 group and significantly decreased after PSMA1 knockdown (Figure 5(a)). Then, CCK-8 results suggested that vector-PSMA1 increased cell viability compared with the control group, and shPSMA1-1# and shPSMA1-2# reduced cell viability in LTEP-s and NCI-H596 cells. Thus, these results demonstrated that upregulated PSMA1 significantly promoted the proliferation of LUSC cells, and PSMA1 downregulation had the opposite effect (Figure 5(b)). A colony formation assay was performed to assess the effect of PSMA1 on colony-forming ability. The number of colonies in the vector-PSMA1 group was significantly increased compared with that in the vector group (negative control), and the shPSMA1-1# and shPSMA1-2# group had significantly decreased colonies compared with the shNC (negative control) group (Figure 2(c)), indicating that the level of PSMA1 was closely associated with the colony-forming ability of LTEP-s and NCI-H596 cells. By examining the cell apoptosis through flow cytometry, the results indicated that the apoptosis of LUSC cells was regulated by the expression of PSMA1 (Figure 2(d)).

## 4. Discussion and Conclusion

LUSC is one main cause of cancer-related mortality all over the word, which was identified to be driven by mutated genes [14]. The therapeutic strategies for LUSC have many obstacles compared with lung adenocarcinoma, in which targeted therapy approaches have been prosperous [15]. Our results revealed that PSMA1 played a pivotal role in LUSC. Recently, several studies revealed that PSMA1 was overexpressed in colon cancer [8] and breast cancer [16], and PSMA1 acted as an oncogene to promote the progression of cancer.

In our study, the result showed that the PSMA1 expression level was notably accumulated in both LUSC patients' tissue and available data based on TCGA dataset. The expression levels of mRNA and protein of PSMA1 were particularly high in clinical tumor tissues compared to normal tissues. These results suggested that PSMA1 might play a role in the development and progression of LUSC. Next, the functions of PSMA1 were explored to uncover the potential mechanism of its action in LUSC.

Patients with LUSC were divided into a PSMA1 low-expression group and PSMA1 high-expression group by the model. The Kaplan-Meier analysis indicated that PSMA1 expression level could be a guide in predicting prognoses and systemic treatments. To further explore the biological function of PSMA1 affecting LUSC processions, the PSMA1 was knocked down and overexpressed in two LUSC cell lines (LTEP-s and NCI-H596) using a lentivirus-mediated shRNA and vector RNA, respectively. Our result demonstrated that PSMA1 overexpression increased the viability and reproduction of tumor cells, suggesting that PSMA1 exerted an oncogenic activity in LUSC procession. Unfortunately, the underlying mechanism of PSMA1 in LUSC was not elucidated in this study, which will be investigated in further studies. It is worth mentioning that collecting more clinical datasets will help to reaffirm the value of PSMA1, which would be in our plans.

In summary, we verified that PSMA1 was overexpressed in LUSC patient's tissues. Functionally, PSMA1 overexpression promoted the growth of LUSC cells by promoting the viability and inhibition of apoptosis of the cells, while PSMA1 knockdown had the opposite effects. In the following research, the investigation would be focused on elucidating the mechanism of PSMA1 in the development of LUSC, which will contribute to comprehensive understanding of tumor progression of LUSC and add the extra direction of therapeutic targets for LUSC.

## Figures and Tables

**Figure 1:** Differentially expressed gene in LUSC based on TCGA database. (a) Volcano plots of differentially expressed gene in the limma package based on an adj.*P*.Val < 0.05 and log |log FC| > 1; (b) volcano plots of differentially expressed gene in the edgR package based on FDR < 0.05 and |log FC| > 1; the red dots represent the upregulated genes; the green dots represent the downregulated genes based; the gray spots represent genes with no significant difference in expression. (c) The Venn diagram demonstrates the intersections of genes between the limma package and edgR package.

**Figure 2:** The prognostic genes in LUSC. (a) The prognostic genes extracted by univariate Cox regression analysis. (b) The trajectory of each prognosis-related candidate gene's coefficient in diffuse-type LUSC was observed in the LASSO coefficient profiles with the changing of the lambda in LASSO algorithm. (c) After the 10-fold cross-validation, a confidence interval was obtained for partial likelihood deviance as the lambda changed. (d) The prognostic genes related with OS extracted by multi-Cox regression analysis.

**Figure 3:** The survival analysis of PSMA1 with LUSC. (a, b) The expression of PSMA1 in tissues from patients with LUSC: (a) TIMER database and (b) UALCAN database. (c, d) The survival analysis of PSMA1 in tissues from patients with LUSC: (c) OS and (d) FP.

**Figure 4:** Analysis of PSMA1 level in cells. (a) The mRNA expression of PSMA1 in tissues of LUSC patients was detected by qRT-PCR. (b) Protein expression of PSMA1 was detected by WB in tissues from patients with LUSC. (c) IHC staining for PSMA1 in tissues of LUSC patients. (d) Quantitative RT-PCR analysis of PSMA1 in LTEP-s, NCI-H596, and NCI-H520 cells. (e) Western blot analysis of PSMA1 in LTEP-s, NCI-H596, and NCI-H520 cells. PSMA1 molecular weight: 84 kDa.

**Figure 5:** The study of the mechanism of PSMA1 in the cell. (a) The protein expression of PSMA1 was analyzed in PSMA1-depleted cells and PSMA1-overexpressed cells by western blot (right) analyses. (b) The viability cell was detected by CCK-8 when PSMA1 was sliced and PSMA1 was overexpressed. The cells were measured at 24, 48, 72, and 96 h. (c) Clone formation assay showing the proliferation ability of the LTEP-s and NCI-H596 cells with the vector-PSMA1 group and shPSMA1-1# and shPSMA1-2# compared with the vector-empty group and shNC group, respectively. (d) Cell apoptosis distribution was determined by flow cytometric analysis in LTEP-s and NCI-H596 cells in the vector-PSMA1 group and shPSMA1-1# and shPSMA1-2# compared with the vector-empty group and shNC group.

**Table 1:** Sequences of shRNAs in the experiment.

Name	Sequence
shRNA-1	GCTGGTTATGATTTTCGAA
shRNA-2	ATTGCTGGTTATGATTTTC
shNC	UUUGUACUACACAAAAGUACUG, CAGUACUUUUGUGUAGUACAAA

**Table 2:** Sequences of primers in the experiment.

Name	Sequence (5′ to 3′)
PSMA1-forward	CAAACTCCCGCAGACTTCTC
PSMA1-reverse	GACCAACTGTGGCTGAACCT
GAPDH-forward	CGCTCTCTGCTCCTCCTGTTC
GAPDH-reverse	ATCCGTTGACTCCGACCTTCAC

**Table 3:** The relationship between the expression level of PSMA1 and the clinicopathological characteristics in LUSC.

Characteristics	Number of patients	PSMA1 Low expression	PSMA1 High expression	*P* value
Number	30	15	15	
Ages (years)				0.713
≤60	13	7	6	
>60	17	8	9	
Gender				0.439
Male	20	9	11	
Female	10	6	4	
TNM stage				0.02^∗^
I	9	8	1	
II	13	4	9	
III	8	3	5	
Pathological grading				0.046^∗^
I	8	7	1	
II	16	6	10	
III	6	2	4	
Smoking				0.065^∗^
Yes	17	6	11	
No	13	9	4	

## Data Availability

All data generated or analyzed during this study are included in this published article.
